The article "Effect of Application of Repeated Downhill Walking Bouts on Ankle Isokinetic Parameters in Children with Obesity" was retracted in 2023. Reasons: signs of a paper mill; compromised peer review; unreliable results or conclusions.

# Effect of Application of Repeated Downhill Walking Bouts on Ankle Isokinetic Parameters in Children with Obesity

**DOI:** 10.1155/2022/1128794

**Published:** 2022-01-28

**Authors:** Hatem H. Allam, Alaa Shafie, Abdulrahman J. Almalki, Dhefallal E. Almalki, Tarek Alsayad, Ahmed M. Alziyadi, Mosfer A. Al-walah, Lamiaa K. Elsayyad

**Affiliations:** ^1^Department of Physical Therapy, College of Applied Medical Sciences, Taif University, P.O. Box 11099, Taif 21944, Saudi Arabia; ^2^Department of Clinical Laboratory Sciences, College of Applied Medical Sciences, Taif University, P.O. Box 11099, Taif 21944, Saudi Arabia; ^3^Department of Medical Rehabilitation and Physiotherapy, Eradah & Mental Health Complex, 2860 Shihar Dist., Taif, Saudi Arabia; ^4^Faculty of Medicine, Al-Azhar University, Cairo, Egypt; ^5^Prince Sultan Hospital, Taif, Saudi Arabia

## Abstract

**Background:**

Obesity among children became of high concern. Obesity can affect many health aspects including muscular strength. Downhill walking is a useful intervention to enhance muscular strength, especially in older adults.

**Objective:**

The current study's purpose was to investigate the effect of repeated bouts of downhill walking on ankle isokinetic parameters in children with obesity.

**Methods:**

32 obese male children aged from 8 to 12 years engaged in the study. The children were divided into two groups: the level walking group (LWG) (*n* = 16) and the downhill walking group (DWG) (*n* = 16). Participants in both groups walked 20 minutes on the treadmill, two sessions per week for 6 weeks, with a speed of 5 km/h, and the treadmill slope used for the DWG was set at –20%. Isokinetic dynamometry (Cybex 6000) was used to analyze the normalized eccentric and concentric torque of both ankle dorsiflexors and plantar flexors of the dominant leg in all participants.

**Results:**

The normalized peak torques for eccentric plantar flexion, concentric plantar flexion, eccentric dorsiflexion, and concentric dorsiflexion significantly increased by 38.66%, 23.87%, 38.58%, and 15.51%, respectively, after repeated bouts of downhill walking. Level walking resulted in nonsignificant improvement in the muscular torques.

**Conclusion:**

Downhill walking is a beneficial intervention in improving ankle muscular torques of obese children.

## 1. Introduction

Obesity was only identified as a health concern affecting adults. More recently, obesity among children became of high concern [1]. Sedentary lifestyles and eating habits are the main factors that result in increased prevalence of obesity among children, for example, spending a long time playing electronic games and eating unhealthy food and sweets [2]. There are many metabolic and psychological problems combined with obesity during early life such as the high risk of type 2 diabetes, early cardiovascular disorders, and low self-esteem. Moreover, it was found that obesity in adulthood was correlated with a high incidence of obesity in the childhood period [3]. The matter is not different in the Kingdom of Saudi Arabia (KSA); the overall prevalence of overweight and obesity in the eastern area of KSA was found to be 19.0% and 23.3%, respectively [4].

Cortney [5] mentioned that the leg muscles have a critical function because they act as the body's shock absorbers. Thus, the strength of the leg muscles, particularly ankle plantar flexors and dorsiflexors, appears to be a critical factor for functional mobility. Furthermore, Ryan [6] stated that the eccentric action of dorsiflexors plays a critical role in ankle stabilization during stance phase while their concentric contraction ensures complete foot clearance during the swing phase. On the other hand, the calf muscles provide the propulsive force for the late stance. Additionally, during the stance phase, the calf muscles control dorsiflexion of the ankle and prevent abnormal pronation so that such activity is eccentric in nature: once the foot strikes the ground, the leg moves forward, and the angle between the foot and the leg decreases which is the dorsiflexion of the ankle [7].

Corbeil et al. [8] reported that obese children have deficits in the ankle muscles' torque required for maintaining stability when they are exposed to any oscillations, so they have a high falling risk. Moreover, McMillan et al. [9] mentioned that the normalized ankle plantar flexor torques were reduced in obese subjects. They reported that obese individuals produce excess hip flexion forces to move the body forward which may indicate weakness of the ankle plantar flexors. Furthermore, Abdelmoula et al. [10] mentioned that obese children have decreased power-related activities that require stability and this may be related to the decreased eccentric torque in the muscles.

Recently, downhill walking has been considered a physical activity that improves functional performance and muscular strength [11]. They added that downhill treadmill walking increases the knee extensor's force by about 5%. Furthermore, Rodio and Fattorini [12] reported that the maximum quadriceps femoris' voluntary contraction was increased after DW in healthy young adults.

Relatively, little is known about the ankle isokinetic parameters in obese children and the effect of repeated downhill walking bouts on these parameters as most studies of DW have concentrated on the knee muscles, with very little mention of ankle muscles. So the children with obesity are in a need for designing specific exercise interventions to improve their muscle strength, functional performance, endurance, and subsequently their daily living activities. So the main aim of this work was to study the effect of repeated downhill walking bouts on ankle isokinetic parameters in these children.

## 2. Methodology

### 2.1. Study Design

The current study was a randomized controlled trial. Initially, a pediatric consultant performed a thorough examination for all children. A double-blind technique was used; the consultant and the participants were not aware of the groups' division. The children were enrolled by calling their guardians. All participants' guardians signed a written informed consent after they were told the full description and aims of the intervention protocol. The study was done at the College of Applied Medical Sciences, Taif University, KSA.

### 2.2. Subjects

A total of 34 obese male children aged from 8 to 12 years were initially selected from the public elementary schools, Taif, KSA, for the study. The G Power program was used to determine the sample size with the following parameters: *α* = 0.05, power 0.90, effect size = 0.6, and Pillai *V* = 0.265. There was attrition of two participants for special circumstances not related to the study; thus, only 32 children completed the experiment. The participants were allocated into two groups using a simple random sampling technique: group I (level walking, LWG, *n* = 16) and group II (downhill walking, DWG, *N* = 16). The inclusion criteria were as follows. All children were right foot dominant. Their body mass index percentile was 95th or more (obese). We had emphasized that all participants did not participate in any type of disciplined intervention during the last 6 months before the beginning of the current work. Additionally, throughout the study period, children were instructed to stay away from any strenuous activities. The participants' accepted score lied between 4 and 7 which is considered mild to moderate activity level. The participants were excluded if they had major musculoskeletal, cardiovascular, or neurological diseases. A flowchart for the study participants is illustrated in Figure 1.

### 2.3. Randomization

A simple random sampling technique was applied to classify the children into the experimental groups. Each child had a random number created using the Excel program, and then, the random numbers from 1 to 16 were selected for LWG while the random numbers from 17 to 32 were selected for DWG.

### 2.4. Leg Dominancy

The following procedures were done to determine the dominant leg: while the participant was standing erect and his legs were parallel to each, he was pushed strongly from behind. The forward-moving leg to restore stability was the dominant one. Moreover, from the same position, the child was asked to kick a ball in front of him, and the leg with which he kicked the ball confirmed the dominant leg.

### 2.5. Physical Activity

The investigator determined the physical activity level through a predesigned questionnaire adopted from Baecke et al. [13]. The score of this questionnaire assesses mutually sport and leisure times. The summation of both values gives the total score for the physical activity level.

### 2.6. Body Mass Index Percentile

The body height and weight were measured by using a stadiometer and Seca 769 digital body weight scale. The children's weight was evaluated while they were unshod. Children's height was assessed in an erect standing position. The data were collected thrice for each variable to avoid errors. BMI was expressed by dividing weight in kilogram on the height in meters squared. To categorize each participant, the BMI percentile was used as the charts of the American Academy of Pediatrics recommended.

### 2.7. Isokinetic Measurements

Isokinetic dynamometry (Cybex 6000) was used to analyze the normalized peak eccentric and concentric torque of both ankle dorsiflexors and plantar flexors of the dominant leg in all participants. The concentric-eccentric mode was used to assess the participants within the range from 10° dorsiflexion to 30° plantar flexion. At first, all children were engaged in 5 minutes of light warming up exercises on a cyclic ergometer (50 to 60 cycles per minute). The following procedures were done to localize the muscle actions: (1) stabilizing straps were put around the waist, thighs, and shoulders, where he was in a semisitting position with the backrest inclined posteriorly 20°. A thigh cuff was used to support the knee in 45° of flexion. (2) The ankle dorsiflexion/plantar flexion attachments for the Cybex 6000 were used as indicated in the manual which supported the foot. (3) The lateral malleolus was in alignment with the device's axis of rotation. (4) The participant was asked to hold his arms crossed over the chest to avoid any synergistic muscle action. (5) The ankle plantar flexion was tested first. (6) The instructions were provided to all children, and they were allowed to take time with the testing equipment to be familiarized with the testing procedures. (7) The angular velocity of 60°/s was used at which children could produce the largest torque compared with higher velocities.

(8) Each participant performed three trials, and the highest one was considered. Each trial consisted of 5 repetitions. The participants had taken one-minute rest after each trial. The children were given verbal reinforcement during every trial to obtain the highest muscular torque [14]. Finally, the preintervention testing was done 6 days before the initial training session, and the postintervention testing was done 3–5 days after the last session to allow adequate time to detect the influence of the intervention on the muscular torque.

### 2.8. Intervention Protocol

Four days prior to intervention, the participants in both groups visited the lab and performed a 5 min walking on the treadmill. This procedure allows participants to be familiarized with all intervention procedures and to protect children in the DWG from potentially damaging DW which will be performed subsequently [15]. Participants in both groups walked 20 minutes on a motorized treadmill, two sessions weekly for 6 weeks, with a speed of 5 km/h, and the treadmill slope used for the DWG and for the LWG was set at –20% and 0%, respectively [12]. All sessions were conducted under the supervision of the study authors.

### 2.9. Ethical Guidelines

The ethical committee, the research and studies department, directorate of health affairs, Taif, KSA, approved the study (ethical approval number 646).

### 2.10. Statistical Analysis

SPSS program version 26 was utilized to analyze the data. The Shapiro-Wilk test, an inspection of Q-Q plots, and Levene's test indicated that the collected data were close to the normal distribution, so parametric analysis was applied. MANOVA and repeated measures ANOVA were used to inspect the demographic data, and repeated measures MANOVA within- and between-subjects effect was used to analyze the study's variables including the ankle plantar flexor and dorsiflexor isokinetic eccentric and concentric peak normalized torque. Regarding the analysis of the demographic data, two tests were used (MANOVA and repeated measures ANOVA). So the alpha level was set at 0.025 while it was 0.05 for the study variables as only one test was used (repeated measures MANOVA).

## 3. Results

### 3.1. Baseline Comparisons

Preintervention, MANOVA, and Bonferroni pairwise comparisons showed nonsignificant differences between LWG and DWG regarding the demographic data (Table 1) and the study variables (eccentric and concentric normalized peak torques for ankle's plantar flexors and dorsiflexors) (Table 2).

### 3.2. Postintervention Comparisons

Repeated measures MANOVA within- and between-subjects effect showed a significant result. The equality of covariance matrices was violated as indicated by Box's test which has had a significant value (*P* = 0.0001) so, Pillai's trace measure was used (Table 3).

### 3.3. Within-Subjects Comparisons

The improvement in LWG was nonsignificant for the four study variables. The normalized peak torques for eccentric plantar flexion, concentric plantar flexion, eccentric dorsiflexion, and concentric dorsiflexion improved by 1.22%, 3.63%, 3.49%, and 3.67%, respectively. On the other hand, the DWG showed a significant improvement. The normalized peak torques for eccentric plantar flexion, concentric plantar flexion, eccentric dorsiflexion, and concentric dorsiflexion increased by 38.66%, 23.87%, 38.58%, and 15.51%, respectively (Table 4). The participants' weight after the intervention for LWG was 55.85 ± 5.45 and for DWG was 57.61 ± 4.29 with nonsignificant changes when it was compared to preintervention (the *P* value for LWG and DWG was 0.62 and 0.34, respectively).

### 3.4. Between-Subjects Comparisons

There was a significant increase in all tested muscular torques of DWG when they were compared to these of LWG postintervention (Table 5).

## 4. Discussion

The purpose of the current study was to investigate the repeated downhill walking bouts' effect on ankle isokinetic parameters among obese children at Taif. This will let us determine an appropriate intervention to improve muscle strength and decrease the incidence of ankle injuries. The normalized peak muscular torques in relation to body weight were used. It is widely used by researchers to remove the confusing effect of the anthropometric factors and precisely indicates the muscular condition [16]. The treadmill parameters were chosen according to Ardigò et al. [17] who reported that the total energy cost of downhill walking at these parameters was minimal.

The study results indicated a significant improvement in the normalized peak muscular eccentric and concentric torque in both plantar flexors and dorsi flexors in the DWG when compared with the baseline and with the LWG. Maeo et al. [18] accorded with these results as they said that the knee extensors' strength was improved even with low-intensity DW for only four sessions, and this improvement was more significant in the eccentric strength. Moreover, Rodio and Fattorini [12] evaluated the effect of DW on strength of the lower limb muscles in teenagers. They said that the knee extensors' peak torque was significantly improved in both dominant and nondominant legs after DW. These findings may be due to the growth and excitement of the powerful fast-twitch fibers stimulated by the DW which are important for the generation of muscular force [12, 19]. Furthermore, Maeo et al. [20] supported our findings when they examined knee extensors' concentric, eccentric, and isometric torque before and after DW. They reported that the knee extension torque was significantly increased after the training period. Additionally, the results obtained by McHugh et al. [21] came in agreement with the current study results. They confirmed that the knee flexors' torque had significantly increased following a low-intensity bout of eccentric exercises. These findings may occur due to improvement in the motor neuron pool to the exercised muscles, the activation of the motor units, improved intermuscular synchronization, and reduced antagonists' activation [21, 22]. Moreover, Vogt and Hoppeler [23] stated that the DW is highly representative of the eccentric contraction that increases the load on the muscles without high effort. So it became essential in strength and endurance programs to enhance performance and prevent injury. They supported the results of the current study when they mentioned that eccentric mode is beneficial to increase muscle strength.

While the cross-sectional area was not evaluated in the present study, the improvement in muscular torque following DW training may be related to the hypertrophy and increase in fiber cross-sectional area that follows this type of training [24]. Further to this, Zoll et al. [25] justified the improved muscular force production after DW to the increase in the IGF-I mRNA growth hormone, which is important for the formation of myofibril protein and stimulation of satellite cells after muscle lengthening contractions.

Moreover, Lynn et al. [26] suggested that the repeated eccentric contraction bouts may induce structural changes in the muscles that may elevate the torque production. One example for these changes is the extra sarcomeres that are serially connected in the muscle after the eccentric training. Additionally, the increase in the muscular torque after the application of repeated eccentric bouts may occur due to the increase in the length of the muscle fascicle which results from the addition of the extra serial sarcomeres to the muscle fibers. The addition of sarcomeres enhances the velocity of muscle contraction leading to more powerful torque production at longer muscle lengths [27, 28, 29].

Furthermore, there was more increase in the eccentric torque than that in the concentric one postintervention. Certain previous studies agreed with this finding. Morgan [30] mentioned that the serially extra sarcomeres connected in the muscle fibers following the eccentric contraction exceeded those produced by concentric training. Furthermore, Maeo et al. [20] reported that the gain in eccentric knee extension torque exceeded that of isometric and concentric after DW training and the justification of this finding was discussed previously. Additionally, Aagaard [31] stated that the muscle activation in untrained subjects is initially decreased during maximal eccentric when compared with maximal concentric contraction. Such reduction is due to the decline in the efferent neural drive. But this inhibition in muscle activation soon faded away when the muscle was engaged in repeated bouts of eccentric training. Blazevich et al. [32] and Vogt and Hoppeler [23] also supported this finding when they reported that the gain in eccentric and isometric strength was doubled after the eccentric training such as DW when compared with the concentric strength.

Concerning LWG, there was an improvement in both normalized eccentric and concentric torque after the intervention, but this improvement was nonsignificant. Rodio and Fattorini [12] agreed with these findings when they compared MVC developed by the quadriceps femoris after level walking (0% inclination), uphill walking (+20% inclination), DW (−20% inclination), and mixed walking on the treadmill. They found that only the DW significantly improved the voluntary contraction without significant improvement in the other walking programs. This may be attributed to the fact that the workload was light and the duration of the training sessions was short to significantly increase the muscular torque.

The alteration in the body composition after the intervention was not significant in any of both groups. This may be due to the fact that the intensity of the exercise program was light to cause significant changes. The total workload (two sessions per week for only six weeks) was low to increase the energy outlay which is supported by Rodio and Fattorini [12].

## 5. Conclusion

The DW resulted in a significant improvement in the normalized muscular eccentric and concentric torque in both plantar flexors and dorsi flexors. Additionally, the improvement in the eccentric torques was more significant than that in the concentric one postintervention. On the other hand, LW improved both eccentric and concentric normalized torque after the intervention, but this improvement was nonsignificant.

## 6. Limitations

There are certain limitations in the current study. Firstly, the female children did not participate in the study because of ethical issues in KSA. Also, the examined isokinetic parameters were only concentric and eccentric torques; other isokinetic parameters, such as power, work, and fatigue, were not considered. Finally, the angular velocity of the current study was 60°/s which is considered as a slow angular velocity, and the results may be different if conducted at higher angular velocities.

## Figures and Tables

**Figure 1:** Flowchart demonstrating the study participants.

**Table 1:** Baseline comparisons for the demographic data.

Variables	LWG (*M* ± SD)	DWG (*M* ± SD)	Mean difference	Sig.
Age (years)	10.53 ± 1.18	10.86 ± 0.96	-0.33	0.39
Weight (kg)	55.81 ± 5.49	57.70 ± 4.44	-1.89	0.29
Height (m)	1.52 ± 0.061	1.56 ± 0.040	-0.031	0.11
BMI	23.97 ± 1.19	23.83 ± 0.87	0.14	0.70
BMI percentile	96.56 ± 1.15	96.19 ± 0.83	0.375	0.30

*M*: mean; SD: standard deviation; Sig.: significance; LWG: level walking group; DWG: downhill walking group.

**Table 2:** Baseline comparisons for the study variables.

Variables	LWG (*M* ± SD)	DWG (*M* ± SD)	Mean difference	Sig.
PNET-plantar (N·m/kg)	1.48 ± 0.15	1.58 ± 0.17	-0.102	0.08
PNCT-plantar (N·m/kg)	1.02 ± 0.19	0.97 ± 0.18	0.047	0.49
PNET-dorsi (N·m/kg)	0.77 ± 0.05	0.80 ± 0.052	-0.026	0.16
PNCT-dorsi (N·m/kg)	0.41 ± 0.056	0.42 ± 0.046	-0.014	0.43

PNET: peak normalized eccentric torque; PNCT: peak normalized concentric torque; *M*: mean; SD: standard deviation; Sig.: significance; LWG: level walking group; DWG: downhill walking group.

**Table 3:** Repeated measures MANOVA within- and between-subjects effect.

Effect		*F*	Sig.
Between subjects	Groups	39.28	0.0001
Within subjects	Time	172.36	0.0001
	Time∗groups	92.26	0.0001

Sig.: significance.

**Table 4:** Bonferroni test for study variables' pairwise comparisons pre-postintervention (within subjects).

	Peak normalized torque (N·m/kg)	Preintervention (*M* ± SD)	Postintervention (*M* ± SD)	Mean difference	Sig.
LWG	Eccentric-plantar	1.48 ± 0.15	1.5 ± 0.15	-0.018	0.27
	Concentric-plantar	1.02 ± 0.19	1.06 ± 0.19	-0.039	0.37
	Eccentric-dorsi	0.77 ± 0.05	0.80 ± 0.05	-0.028	0.37
	Concentric-dorsi	0.41 ± 0.056	0.42 ± 0.06	-0.016	0.11

DWG	Eccentric-plantar	1.58 ± 0.17	2.19 ± 0.16	-0.61	0.0001
	Concentric-plantar	0.97 ± 0.18	1.2 ± 0.1	-0.23	0.0001
	Eccentric-dorsi	0.80 ± 0.052	1.1 ± 0.16	-0.30	0.0001
	Concentric-dorsi	0.42 ± 0.046	0.49 ± 0.08	-0.07	0.0001

*M*: mean; SD: standard deviation; Sig.: significance; LWG: level walking group; DWG: downhill walking group.

**Table 5:** Bonferroni test for the study variables' pairwise comparisons postintervention (between subjects).

Peak normalized torque (N·m/kg)	LWG (*M* ± SD)	DWG (*M* ± SD)	Mean difference	Sig.
Eccentric-plantar	1.5 ± 0.15	2.19 ± 0.16	-0.69	0.0001
Concentric-plantar	1.06 ± 0.19	1.2 ± 0.1	-0.15	0.008
Eccentric-dorsi	0.80 ± 0.05	1.1 ± 0.16	-0.30	0.0001
Concentric-dorsi	0.42 ± 0.06	0.49 ± 0.08	-0.06	0.018

*M*: mean; SD: standard deviation; Sig.: significance; LWG: level walking group; DWG: downhill walking group.

## Data Availability

The authors will provide the data that support the conclusion if requested.
